RETRACTED

# Antioxidant, Anticancer, and PXR-Dependent CYP_3_A_4_ Attributes of *Schweinfurthia papilionacea* (Burm.f.) Boiss., *Tricholepis glaberrima* DC. and *Viola stocksii* Boiss

**DOI:** 10.1155/2022/9366223

**Published:** 2022-02-16

**Authors:** Amir Shahbaz, Javed Iqbal, Banzeer Ahsan Abbasi, Wasim Akhtar, Iram Fatima, Syeda Anber Zahra, Sobia Kanwal, Javad Sharifi-Rad, Hassan Sher, Tariq Mahmood, William C. Cho

**Affiliations:** ^1^Department of Plant Sciences, Faculty of Biological Sciences, Quaid-i-Azam University, Islamabad 45320, Pakistan; ^2^Department of Botany, Bacha Khan University, Charsadda, Khyber Pakhtunkhwa, Pakistan; ^3^Department of Botany, University of Azad Jammu and Kashmir, Muzaffarabad, Pakistan; ^4^Department of Biotechnology, Fatima Jinnah Women University, Rawalpindi, Pakistan; ^5^Department of Biology and Environmental Sciences, Allama Iqbal Open University, Islamabad, Pakistan; ^6^Facultad de Medicina, Universidad del Azuay, Cuenca, Ecuador; ^7^Center for Plant Sciences and Biodiversity, University of Swat, Kanju 19201, Pakistan; ^8^Department of Clinical Oncology, Queen Elizabeth Hospital, Kowloon, Hong Kong

## Abstract

Present study established the biological potential of *Schweinfurthia papilionacea*, *Tricholepis glaberrima* and *Viola stocksii* extracts for their potential applications in drug formulations. Initially, FTIR was performed to ascertain functional groups and then plant extracts were prepared using five solvents depending on the polarity. Total phenolic contents were observed in the range of 36.36 ± 1.08 mg GAE/g to 95.55 ± 2.46 mg GAE/g while flavonoid contents were found in the range of 10.51 ± 0.25 mg QE/g to 22.17 ± 1.79 mg QE/g. Antioxidant activity was determined using TRP, CUPRAC, TAC and DPPH assays and was recorded highest in *S. papilionacea* followed by *T. glaberrima* extracts. TPC and TFC were found to be strongly correlated with TRP (r > 0.50), CUPRAC (r > 0.53) and DPPH (r = 0.31 and 0.72) assay while weakly correlated with TAC (r = 0.08 and 0.03) as determined by Pearson correlation analysis. Anticancer activity showed that *S. papilionacea* chloroform extracts possess highest cell viability (85.04 ± 4.24%) against HepG2 cell lines while *T. glaberrima* chloroform extracts exhibited highest activity (82.80 ± 2.68%) against HT144 cell lines. Afterwards, highest PXR activation was observed in *T. glaberrima* (3.49 ± 0.34 *μ*g/mL fold) at 60 *μ*g/mL and was correlated with increase in CYP_3_A_4_ activity (15.0 ± 3.00 *μ*g/mL IC_50_ value). Furthermore, antimalarial activity revealed >47600 IC_50_ value against *P. falciparum* D6 and *P. falciparum* W2 and antimicrobial assay indicated highest activity (32 ± 2.80 mm) in *S. papilionacea* against *C. neoformans*. At the end, GC-MS analysis of n-hexane plant extracts showed 99.104% of total identified compounds in *T. glaberrima* and 94.31% in *V. stocksii*. In conclusion, present study provides insight about the different biological potentials of *S. papilionacea* and *T. glaberrima* extracts that rationalize the applications of these extracts in functional foods and herbal drugs for the management of oxidative-stress related diseases, antimicrobial infections and liver and skin cancer.

RETRACTED

## 1. Introduction

Now-a-days, use of herbal medicines has considerably increased worldwide in both developing and industrialized countries [1] owing to the fact that many practitioners recommend these plant-based products or complementary medicines on the basis of their chemical free nature and more reliable results [2, 3]. Till now, more than 53,000 species have been reported to be utilized for health purposes [4] and trade market of medicinal drugs is almost US $60 billion which is continuously rising at a rate of 7% per annum [5]. Plant-based crude drugs consist of various bioactive compounds that are involved in curing diseases. Among these, phenolics and flavonoids are predominantly considered as effective free radical scavengers and exhibit antimicrobial and anticancer properties [6, 7].

Phenolic compounds exhibit antioxidant potential due to donation of hydrogen atom and electron to free radicals causing the break of chain reaction of oxidation. The antioxidant effect depends on the number and position of hydroxyl groups [6]. Phenolic compounds such as hydroxybenzoic acids (sinapic acid, ellagic acid) and hydroxycinnamic acids (p-coumaric acid) derived from various fruits and vegetables function as potent anticancer agents [8–10]. Despite numerous studies on phenolic compounds and plant extracts, the exact relationship between anticancer and antioxidant activity needs to be studied more comprehensively. Flavonoids disrupt the electron transport chain due to their radical scavenging properties and chelate metal ions [11]. Hyun et al. [12] observed that free radical scavenging effect increases with increase in the number of hydroxyl groups in the flavonoid molecule.

The antioxidant activity of hydroxyflavones depends on the number of hydroxyl groups and their position in the molecule and thus, dihydroxyflavones are considered as strong antioxidants [11]. Similarly, hydroxyflavones along with many other flavonoid compounds like apigenin, kaempferol, naringin, anthocyanins, luteolin and catechin obtained from plants are known for antioxidant activity and have significant impact on melanoma, oesophageal and breast carcinomas due to their low toxicity effects and ability to interact with DNA [9, 13–15]. Moreover, flavopiridol is a synthetic derivative, similar to flavonoids, and exhibit effect on cyclin-dependent kinases [16]. These examples prove the importance of natural compounds *i.e.* phenolic and flavonoid compounds in the development of new drugs.

RETRACTED

These phytochemicals exist in most of the plant species in free and bound forms and are safe for consumption as dietary supplements [17, 18]. Several studies have revealed that disease preventive potential of plant-based food is correlated with polyphenol constituents present in medicinal plants [19]. Overproduction of reactive oxygen species lead to degenerative diseases such as diabetes, heart diseases and aging [20]. Recent studies showed that, in addition to the antimicrobial activities, these compounds exhibit diverse molecular and biochemical functions in plant such as signaling, mediating auxin transport, and plant defense [21, 22]. Numerous synthetic antioxidants are used in industries for scavenging free radicals, however, their application is restricted due to their toxicity and deleterious side effects [23].

This unique property of plant-based drugs act as a paramount in the development of medicines for various diseases like cancer and diabetes [6, 7]. About 18.1 million cancer cases and 19.6 million cancer-related deaths were reported in 2018 and 17 million cases were recorded during 2020 [24]. Lung cancer and breast cancer are the major cause of cancer occurring worldwide and the later one is commonly detected in women [25]. Chemicals and radiation-based treatments are applied in cancer therapy but high proportion of treatment failure is still a major issue [26, 27]. Due to the alarming increase in the cancer incidents, greener and eco-friendly approaches should be implemented for the synthesis of anti-cancer drugs [28, 29].

CYP_3_A_4_ belongs to the cytochrome P450 (CYP) family of enzymes that is specifically involved in the metabolism of xenobiotics and endogenous compounds [30]. CYP_3_A_4_ expression is induced *in vivo* as well as *in vitro* in response to the xenobiotics (like rifampicin) and medicinal plants for example *Mitragyna speciosa*, *Dodonaea angustifolia* and *Euphorbia tirucalli* [31, 32]. Pregnane X receptor (PXR) (or pregnane-activated receptor) chiefly aids in regulating gene expression of CYP_3_A_4_ [33]. Although PXR itself is activated by xenobiotics and phytochemicals like hyperforin from *Hypericum perforatum* [34]. PXR along with its target genes play key role in regulating physiological functions and homeostasis such as artemisinin (*Artemisia annua*) is known as the activator of PXR and helps in preventing severity of chronic inflammatory bowel disease by expressing CYP_3_A_4_ enzyme [35, 36].

RETRACTED

Despite the plethora of literature on innumerable species, many plants still need to be explored. *S. papilionacea* (family Scrophulariaceae) grows under extreme hot conditions [37] and is used to promote diuresis, cure fever and diabetes [38, 39]. *T. glaberrima* belongs to family *Asteraceae* and is used by ancient healers as aphrodisiac, liver disorders, inflammation and antidepressant [40, 41]. However, *V. stocksii* is a member of family *Violaceae* which consists of only one genus and 17 species specifically growing in Pakistan [42]. Hence, preliminary studies were aimed to determine the functional groups, bioactive compounds and biological potential of *S. papilionacea, T. glaberrima* and *V. stocksii* so that they could be used as natural source of medication with potential application in industries.

## 2. Materials and Methods

### 2.1. Plant Collection and Extracts Preparation

*S. papilionacea, T. glaberrima* and *V. stocksii* were collected from Dera Ghazi Khan (Pakistan) in 2018 and their aerial parts were washed, shade-dried, powdered and then extracted with five solvents *viz.* methanol, ethanol, ethyl acetate, chloroform and n-hexane (35 g in 350 mL each) for three days. Subsequently, extracts were filtered using Whatmann filter paper no. 1 followed by evaporation using rotary evaporator. Obtained crude extracts were stored at 4°C for experimental analysis.

### 2.2. Identification of Functional Groups Using FTIR

Perkin Elmer- Frontier FTIR spectrometer (model 65) was used to determine various functional groups in the three plant species. Plants were dried, powdered (10 mg) and added in 100 mg of dried potassium bromide and pellet was formed. Subsequently, 5 x 106 Pa pressure was applied to these pellets in an evacuated dye and then the spectras were observed at 4000 – 400 cm^−1^ frequency [43].

### 2.3. Total Phenolic and Flavonoids

Initially, 6% sodium carbonate solution was prepared by adding 6 g of sodium carbonate in 100 mL of distilled water and folin-ciocalteu reagent was made in 90 mL of distilled water. Then, total phenolic content (TPC) was determined by adding gallic acid in Folin-ciocalteu reagent (90 *μ*L) and sodium carbonate (90 *μ*L) and calibration curve was made. Then, plant extracts (20 *μ*L) were added in the same reagent and the absorbance was recorded at 630 nm. Total flavonoid content (TFC) was determined using aluminum chloride calorimetric method. For this, stock solution of 10% aluminum chloride was made by adding 10 g of aluminum chloride in 100 mL of distilled water and 1 M of potassium acetate was made by dissolving 98.15 g of potassium acetate in 1 L of distilled water. Subsequently, 10 *μ*L of aluminum chloride was added in to 20 *μ*L of plant extract, 10 *μ*L of potassium acetate and 160 *μ*L of distilled water and placed for incubation (30 minutes). The absorbance was recorded at 415 nm and results were expressed as mg QE/g sample [44].

RETRACTED

### 2.4. Determination of Antioxidant Assays

#### 2.4.1. Total reducing power (TRP) assay

Each plant extract (200 *μ*L) was dissolved in the phosphate buffer (500 *μ*L) and potassium ferricyanide (500 *μ*L) followed by incubation at 50°C. After 20 minutes, Trichloroacetic acid (TCA) (500 *μ*L) was added and then centrifuged for 10 minutes to collect the supernatant. Then 0.1% ferric chloride (100 *μ*L) was mixed in the supernatant and the absorbance was recorded at 630 nm [45].

#### 2.4.2. Cupric Ions Reducing Antioxidant Capacity (CUPRAC) Assay

Initially, 0.01 M CuCl2 solution was prepared by adding 0.42 g of CuCl_2_ in 100 mL of water and then diluted to 250 mL. Then, 7.5 mM ethanol neocuproine (Nc) solution was made by dissolving 0.039 g of Nc in ethanol and 1 M ammonium acetate buffer solution was prepared by adding 19.27 g of ammonium acetate in 1 L of distilled water (pH 7.0). Afterwards, 10 *μ*L of CuCl_2_ solution, 10 *μ*L of ammonium acetate and 10 *μ*L of ethanol neocuproine were mixed with 20 *μ*L of each extract and the volume was adjusted to 1 mL by adding distilled water. After 30 minutes, absorbance was measured at 515 nm [46].

#### 2.4.3. Total Antioxidant Capacity (TAC)

To determine the antioxidant potentials, 28 mM sodium phosphate (1.68 g), 4 mM ammonium molybdate (0.25 g) and sulphuric acid (1.63 mL) were dissolved in 50 mL of distilled water to prepare reaction mixture. Then each plant extract (50 *μ*L) was added in the reaction mixture followed by the incubation at 95°C and then absorbance was noted at 630 nm [47].

#### 2.4.4. DPPH Scavenging Assay

DPPH (3.9 mg) was added in methanol (100 mL) and then incubated for 30 minutes in dark. Three different concentrations of plant extracts (10, 20 and 40 *μ*L) were added in DPPH solution (180 *μ*L) and absorbance was measured spectrophotometrically after 60 minutes. Ascorbic acid was used as a standard and percentage inhibition and IC_50_ values were calculated [48]:

(1) $$\begin{array}{c} \text{Percentage scavenging activity}=\text{Ab}{\text{s}}_{\text{control}}–\text{Ab}{\text{s}}_{\text{sample}}/\text{Ab}{\text{s}}_{\text{control}}\times 100 \end{array}$$

### 2.5. Anticancer Assay

HepG2 (liver cancer), HT144 (skin cancer) cell lines were grown in DMEM augmented with 10 percent FBS along with 1 percent antimycotic (ABAM) and maintained in a tissue culture cabinet under 37°C conditions with 95 percent air and 5 percent CO_2_ (Manassas, VA, United States). MTT (3-(4,5-dimethylthiazol-2-yl)-2,5-diphenyl-2H-tetrazolium bromide) assay was carried out to detect the inhibitory effect of selected methanolic, ethanolic, ethyl acetate and chloroform extracts on HepG2 (liver cancer) and HT144 (skin cancer) cell line. The reactant cell lines were held for 24 h at a density of 5 × 10^4^ cells per well in 96-well plates followed by addition of plant extracts. Media were subsequently extracted and 5 mg/mL of MTT reagents were loaded along with sterile PBS followed by 4 h incubation. In addition, MTT solution was extracted and DMSO was used to dissolve precipitate formazan. Finally, absorbance was measured at 570 nm.

RETRACTED

### 2.6. PXR-Mediated CYP_3_A_4_ Induction by Luciferase Reporter Assay

The pSG5-hPXR plasmid was obtained from Southwestern Medical Center, University of Texas [49] and PCR5 (CYP_3_A_4_-PXR response element-LUC comprising of 0/-362 proximal and 7208/7797 distal PXR response element regions fused upstream of luciferase) was taken from the University of Sydney [50]. PXR activation by the methanolic plant extracts was evaluated in cancer cell lines transfected with both plasmid DNA (25 *μ*g each) by electroporation [51]. About 50,000 cells per well seeding density was used and after 24 h plant extracts and positive control were added at different concentrations (6.7, 20 and 60 *μ*g/mL for extracts and 1.1, 3.3 and 10 *μ*M for positive control). Subsequently, 40 *μ*L of luciferase reagent was added in each well and luminescence was recorded on Spectramax plate reader (Sunnyvale, USA). Ketoconazole was used as a positive control for CYP_3_A_4_ inhibition and rifampicin was used as a positive control for PXR assay. At the end, fold induction was determined in the treated cells in comparison to the control.

### 2.7. Antimalarial Lactate Dehydrogenase Assay

LDH assay was conducted as it is an effective diagnostic test for malaria with a sensitivity for *P. falciparum* detection ranging from 94% to 95% and *in vitro* test is easy in comparison to the tests performed on human beings. Briefly, two *Plasmodium falciparum* clones namely chloroquinone-sensitive (CS) Sierra Leone D6 and chloroquinone-resistant (CR) Indochina W2 were used. Plant extracts were prepared in DMSO at different concentrations ranging from 47600 – 5288.9 ng/mL and added to the *P. falciparum* cultures (2% haematocrit, 2% parasitaemia) in the 96 -well plates. Afterwards, these plates were placed in the humidified chamber containing 90% N_2_, 5% CO_2_ and 5% O_2_ and were incubated (37°C) for 48-120 hours. Growth of parasites was ascertained by using Malstat reagent and chloroquinone was used as a standard [52]. IC_50_ values were observed by the dose-response analysis and selectivity indices (SI) were obtained by measuring the cytotoxicity of extracts on mammalian cells (VERO; monkey kidney fibroblast).

RETRACTED

### 2.8. Antimicrobial Assay

As the methanol extracts of all plants displayed highest antioxidant and anticancer activities, so these were selected further to examine the antimicrobial potential of plants against five bacterial strains *viz. Escherichia coli*, vancomycin-resistant *Enterococcus faecium*, methicillin-resistant *Staphylococcus aureus, Klebsiella pneumoniae* and *Pseudomonas aeruginosa* and three fungal species including *Cryptococcus neoformans*, *Candida albicans* and *Aspergillus fumigatus* by using agar disc diffusion assay [53]. Bacterial strains were cultured in nutrient broth medium at 37°C while the fungal strains were sub-cultured using SDA media at 25°C. Each methanolic plant extract was tested using 200 *μ*g/mL concentration and oxytetracycline and chloramphenicol were used as standards. In the end, inhibition zones were measured with the help of ruler in millimeters.

### 2.9. GC-MS Analysis

Initially, 1 g of each plant powder prepared from aerial parts was sonicated in 4 mL of n-hexane for 1 hour and then supernatant was filtered using Millex- GV (0.22 *μ*m). Samples were examined using Agilent 7890 GC instrument equipped with Agilent 7693 auto-sampler and Agilent 5975 mass specific detector. A fused silica capillary column coated with 0.25 *μ*m film of 5% phenyl methyl silicone (HP- 5MS) was used with helium as carrier gas at 1 mL/min flow rate. The oven was held for 2 min at 45°C and then programmed at 1.5°C/min to 100°C and 2°C/min to 200°C. About 1 *μ*L of sample was introduced in split mode (10 : 1) with 82.7 kPa pressure in the column. The injector temperature was set at 250°C and ion-source temperature was adjusted at 280°C. Mass spectra were noted at 70 eV from 40 to 550 m/z and scanning speed was set at 1666. Total GC running time was almost 30 minutes and compounds were recognized by comparing spectra with Wiley and NIST databases. Finally, relative percentage was ascertained by comparing peak area with total area.

### 2.10. Statistical Analysis

All data represents mean ± standard error and ANOVA was performed using statistix version 8.1 to compare mean values by using LSD. Pearson correlation analysis was performed using Microsoft Excel and IC_50_ values were calculated by graphpad prism [54].

## 3. Results

### 3.1. FTIR Analysis

FTIR spectra indicated the presence of various functional groups by producing strong, medium and narrow peak intensities at 3438.90 cm^−1^ to 519.04 cm^−1^ frequency. The band detected at ~3296 cm^−1^ could be related to the OH-bending vibration whereas band found at ~2900 cm^−1^ might be due to C-H stretch. Bands detected at ~1662 cm^−1^ showed the presence of C=C stretch (alkenes) while bands observed at ~1015 cm^−1^ could be related to the occurrence of C-O stretching vibration. Some bands were also identified at <600 cm^−1^ relating to the alkyl halides (C-Br, C-Cl stretch) as presented in Figure 1. Most of the functional groups were commonly present in all species such as alkanes (C-H stretch), alcohols and phenols (O-H stretch), alkyl halides (C-Br, C-Cl stretch), carboxylic acids, esters and ethers (C-O stretch). However, alkenes (-C=C stretch) were absent in *T. glaberrima* and were detected in *S. papilionacea* and *V. stocksii*. Likewise, 1° amines (N-H bend) were observed in *T. glaberrima* instead of aliphatic amines (C-N stretch) that were recorded in other species. Moreover, peaks of C-C stretch and N-O stretch were only detected in *V. stocksii* showing the existence of aromatics and nitro compounds which were lacking in other species.

RETRACTED

### 3.2. Determination of TPC and TFC

Results revealed highest phenolic contents in the methanolic and chloroform extracts of *S. papilionacea* (95.55 ± 2.46 mg GAE/g and 86.26 ± 2.90 mg GAE/g) while lowest TPC was recorded in the n-hexane extracts of *S. papilionacea* and *V. stocksii* (36.36 ± 1.08 mg GAE/g and 50.281 ± 3.32 mg GAE/g). However, *S. papilionacea* ethanolic extract and *V. stocksii* methanolic extract revealed highest TFC (22.17 ± 1.79 mg QE/g and 22.05 ± 1.96 mg QE/g) and the ethyl acetate extracts of *S. papilionacea* and *T. glaberrima* showed lowest flavonoid contents (10.51 ± 0.25 mg QE/g and 11.61 ± 0.29 mg QE/g). Overall, TPC was found in decreasing order of methanolic extracts > chloroform extracts > ethanolic extracts > ethyl acetate extracts > n-hexane extracts while TFC was observed in descending order of methanolic extracts > ethanolic extracts > chloroform extracts > n-hexane extracts > ethyl acetate extracts (Figure 2).

### 3.3. Antioxidant Assays

Antioxidant activity of selected species was confirmed by four assays namely TRP, CUPRAC assay, TAC and DPPH assay. Highest reducing power (> 0.4 absorbance) was observed in the ethanolic and methanolic extracts while extracts prepared in all other solvents showed lowest activity. Among plants, activity was found in descending order of *S. papilionacea* > *T. glaberrima* > *V. stocksii* (Figure 3(a)). In case of CUPRAC assay, *S. papilionacea* showed activity in the range of 6.60 ± 0.48 mg/g (n-hexane extract) to 61.28 ± 1.57 mg/g (methanolic extract) and in *T. glaberrima* it was found in the range of 7.34 ± 0.48 mg/g (n-hexane extract) to 56.50 ± 0.70 (methanolic extract). However, among all species *V. stocksii* revealed lowest CUPRAC activity ranging from 6.77 ± 0.84 mg/g (n-hexane extract) to 40.94 ± 0.37 mg/g (methanolic extract), respectively (Figure 3(b)).

RETRACTED

Total antioxidant capacity was detected highest in the methanolic and ethyl acetate extracts of *S. papilionacea* (59.30 ± 1.42 mg/g and 56.53 ± 1.42 mg/g) and lowest in the ethyl acetate extracts of *V. stocksii* (15.08 ± 1.34 mg/g) and n-hexane extracts of *T. glaberrima* (19.62 ± 0.24 mg/g) (Figure 3(c)). In general, methanolic and chloroform extracts showed highest TRP, CURAC and TAC, hence these extracts were further selected to ascertain DPPH activity of selected species. DPPH activity was performed at five concentrations to determine IC_50_ value and ascorbic acid (standard) displayed IC_50_ value of 296.10 *μ*g/mL. Results revealed that methanolic extracts exhibited highest DPPH activity (IC_50_< 600 *μ*g/mL) as compared to the chloroform extracts. Among all species, *S. papilionacea* methanolic extract revealed highest scavenging activity (IC_50_ value: 322.90 *μ*g/mL) followed by *T. glaberrima* methanolic extract (IC_50_ value: 564.10 *μ*g/mL). Pearson correlation analysis of DPPH assay with respect to TPC and TFC indicated moderately strong relationship with TPC (r = 0.31) and highly positive correlation with TFC (r = 0.72) (Figure 3(d) and 4(d)). Contrarily, Pearson correlation analysis revealed strongly positive relationship of selected phytochemicals with TRP (r > 0.50) and with CUPRAC (r > 0.53) assay while weak correlation was detected when TAC was analyzed with phenolic (r = 0.08) and flavonoid contents (r = 0.03) (Figures 4(a)to 4(c)).

### 3.4. Anticancer Assay

Results revealed that chloroform extracts of *S. papilionacea* and *T. glaberrima* exhibited highest cell viability (85.04 ± 4.24% and 77.45 ± 4.24%) against liver cancer (HepG2) cell line. In case of HT144 (skin cancer) cell line, chloroform, ethyl acetate and ethanolic extracts of *T. glaberrima* indicated highest activity (82.8 ± 2.68%, 75.97 ± 2.85% and 75.89 ± 1.41%) as compared to the *S. papilionacea* and *V. stocksii* extracts. Doxorubicin was used as a standard which showed 96.58 ± 3.05% cell viability against HepG2 and 93.73 ± 6.74% against HT144 (Figures 5(a) and 5(b)). Pearson correlation of anticancer assays indicated strongly positive correlation with the phenolic compounds (r > 0.61) while both anticancer activities were negatively correlated with the flavonoids contents (r < -0.03) as shown in Figures 5(c) and 5(d).

RETRACTED

### 3.5. Luciferase Reporter Gene Assay

In this assay, three different concentrations (6.7, 20 and 60 *μ*g/mL) were used to observe the fold induction of PXR and rifampicin was used as a standard inducer. The comparative fold-induction of CYP_3_A_4_ revealed that *T. glaberrima* (3.49 ± 0.34 *μ*g/mL fold; 15.00 ± 3.00 *μ*g/mL IC_50_ value) was found to be highly effective in inducing CYP_3_A_4_, followed by *V. stocksii* (2.70 ± 0.42 *μ*g/mL fold; 26.5 ± 1.50 *μ*g/mL IC_50_ value) and *S. papilionacea* (2.29 ± 0.20 *μ*g/mL fold; 27.50 ± 0.50 *μ*g/mL IC_50_ value) as shown in Table 1. Moreover, none of the samples were revealed cytotoxic up to 100 *μ*g/mL.

### 3.6. Antimalarial Assay

Results revealed that all the plant extracts were found to be insignificant when tested against *P. falciparum* clones as they showed IC_50_ value greater than 47600 (Table 2).

### 3.7. Antimicrobial Assay

Antibacterial activity of methanolic extracts was tested against five strains which revealed highest activity in *T. glaberrima* against vancomycin-resistant *E. faecium* (11 ± 1.4 mm) followed by *V. stocksii* against *E. coli* (10 ± 0.7 mm). *T. glaberrima* and *S. papilionacea* showed average activity against *E. coli* (9 ± 0 mm and 8 ± 2.8 mm) while *V. stocksii* exhibited lowest activity against *E. faecium* (2 ± 0 mm). However, selected plant extracts revealed insignificant activity against *P. aeruginosa*, *K. pneumoniae* and methicillin-resistant *S. aureus* as no zone of inhibition was observed against them. In case of antifungal assay, inhibition zones were detected in decreasing order of *C. neoformans* > *C. albicans* > *A. fumigatus*. Overall, all plant extracts were found to be highly active against fungal species as compared to the bacterial species (Table 3).

### 3.8. Metabolomic Profiling of T. glaberrima and V. stocksii

GC-MS analysis confirmed the existence of 15 compounds in *T. glaberrima* and 17 compounds in *V. stocksii* including hydrocarbons, fatty acids and alcohols that were eluted at different retention times (Figure 6). Heptane was detected at the lowest retention time (7.18 min) in both species *i.e.* 0.57% in *T. glaberrima* and 1.17% in *V. stocksii.* However, all other compounds were observed at the retention time greater than 46.24 min. In *T. glaberrima*, Eicosane was found in highest concentration (44.60%) at 76.70 min and 69.77 min followed by Neophytodiene (13.22%) at 46.40 min whereas all other remaining compounds were present in lowest concentration *i.e.* < 6%. On the contrary, 9,12-octadecadienoic acid (Z, Z)- was found to be present in highest concentration (40.965%) at 52.91 and 53.08 min in *V. stocksii*, followed by n-Hexadecanoic acid (16.09%) at 48.90 min.

RETRACTED

Most of the compounds were present in both species except few compounds such as Hexadecane (0.81%), 1-Tridecyne (3.95%) and Eicosane (44.60%) were only found in *T. glaberrima* while tetracosane (5.24%), 3-Eicosyne (1.51%), Dibutyl phthalate (0.65%), Bis(2-ethylhexyl) phthalate (1.23%) were only observed in *V. stocksii*. Overall, *T. glaberrima* exhibited highest concentration of compounds *i.e.* 99.10% as compared to the *V. stocksii* which displayed 94.31% compounds. Various compounds isolated at different retention times along with their molecular weight and concentration is presented in Table 4.

## 4. Discussion

*S. papilionacea*, *T. glaberrima* and *V. stocksii* are well recognized for their diverse ethnobotanical uses [38, 40, 41], however, very few studies are available regarding their biological and biochemical properties which is essential for their application in traditional and modern medicines. Henceforth, in the present work, extracts of selected species were prepared using two polar (methanol and ethanol), one slightly polar (ethyl acetate) and two non-polar (chloroform and n-hexane) solvents systematically and then biological assays were conducted using standard protocols. Initially, FTIR analysis was carried out to observe the presence of various alkanes, alcohols, phenols, alkyl halides, carboxylic acids and ethers in the selected species as it is a simple analytical tool used to determine different functional groups of the compounds existing in the medicinal plants [55].

Plant extracts contain important secondary metabolites such as alkaloids, terpenoids, phenolics and flavonoids which exhibit crucial ecological and biological functions in plants [56]. Polyphenols including flavonoids are well-known non-enzymatic antioxidants that can neutralize free radicals. The quantity and composition of plant-derived phenolic products used as food and medicine are also important as antioxidants and have a great impact in human diet and health [7]. Present study revealed that methanolic extract of *S. papilionacea* and *T. glaberrima* exhibited highest TPC *i.e.* 95.55 ± 2.46 mg GAE/g and 80.55 ± 1.61 mg GAE/g among all polar extracts while *S. papilionacea* and *T. glaberrima* chloroform extracts displayed highest phenolic contents *i.e.* 86.26 ± 2.90 mg GAE/g and 80.55 ± 0.91 mg GAE/g among non-polar extracts. Subsequently, three antioxidant assays namely TRP, CUPRAC and TAC were performed to investigate the antioxidant potential of these extracts as these assays chiefly serve as an indicator of the antioxidant potential.

Our results revealed that all extracts possess antioxidant activity in each of the assays, but the polar (methanolic and ethanolic) extracts exhibited highest reducing power and cupric ions antioxidant capacity in comparison to the other extracts. Moreover, TAC was observed highest in the methanolic and chloroform extracts. Hence, the methanolic and chloroform extracts were further examined to ascertain DPPH activity of selected species. Comparatively, DPPH activity was also observed in descending order of *S. papilionacea* > *T. glaberrima* > *V. stocksii* in both extracts. Our study approves former research work of Ahmed et al. [57] indicating lowest antioxidant potential in *V. stocksii* extracts. Pearson correlation analysis further confirmed that antioxidant potential is directly correlated with the presence of phenolic and flavonoid compounds. These antioxidant assays provide a basis and rationale for exploiting these extracts as standardized antioxidant ingredients in various foods, nutraceuticals and dietary supplement industries.

RETRACTED

Present study also correlates with the earlier findings indicating that the extracts which possess high polarity components mainly contribute to the antioxidant power of medicinal plants [58]. Previously, Khasawneh et al. [59] reported that *S. papilionacea* ethanolic extract exhibit 127.40 *μ*g/mL (IC_50_ value) DPPH scavenging activity. Similarly, Naphade et al. [60] also determined the antioxidant activity in the methanol, chloroform and aqueous extracts of *T. glaberrima* by using different assays namely ferric thiocyanate (FTC) and thiobarbituric acid (TBA) assay. However, no other detail study is available on the antioxidant potential of the selected medicinal plants so far. Besides, previous reports complement similar results that plant extracts rich in phenolic compounds possess strong antioxidant activity [61]. Hence, it can be concluded that higher radical scavenging activity is due to the presence of these phenolic compounds [62].

Antioxidants are also known to exhibit key role in preventing cancer by neutralizing the lethal effects caused by the reactive oxygen species [63]. Variations in CYP_3_A_4_ gene expression through the nuclear receptors such as PXR is considered as a leading cause of drug-unresponsiveness and toxicity [31]. In present study, selected extracts were found to be more active against HT144 cell line owing to the existence of phenolic compounds as determined by PCA. Subsequently, reporter gene assay revealed highest PXR activation potential in *T. glaberrima* (3.49 ± 0.34 *μ*g/mL fold) at 60 *μ*g/mL that was associated with an increase mRNA expression and ultimately in the activity of CYP_3_A_4_ (15.00 ± 3.00 *μ*g/mL IC_50_ value). Large-scale production of the desired secondary metabolites by metabolic engineering tools can be used to overwhelm the bioactive compounds availability limitations from medicinal plants and to improve the productivity beneficial from both bioprocessing and molecular farming [56]. Previously, Maqsood et al. [64] reported that *S. papilionacea* methanolic extract possess 70% viability in *Artemesia scoparia* after 24 h treatment and 7% viability in rhabdomyosarcoma (RD) cell lines at 48 h treatment, hence indicating the cytotoxic potential of plant extract. Therefore, it can be suggested that *in vivo* studies should be executed in future, to validate the cytotoxic potential of these extracts at various concentrations. The observed antioxidant and anticancer activities in this study justified the traditional use of *S. papilionacea* and *T. glaberrima* for therapeutic purposes.

RETRACTED

Malaria is also one of the major causes of health problem occurring globally and leads to the increase number of deaths annually [65]. The resistance of the *P. falciparum* to the synthetic drugs has increased the requisite of novel antimalarial products [66]. Present study revealed that selected extracts were ineffective (IC_50_ value >47600) against *P. falciparum* D6 and *P. falciparum* W2 and thus, could not be recommended to be utilized in preparing antimalarial drugs. So far, this is the first report on the antimalarial activity of selected species.

Various polyphenol-rich formulations are also known to treat different microbial diseases such as Huangchin is an herbal formulation used for the infected oral wounds [67]. In current study, all extracts moderately reduced the growth *E. coli* and vancomycin-resistant *E. faecium*. However, in case of antifungal assay, extracts were found to be highly active against *C. neoformans i.e.* inhibition zones ranged from 22 ± 1.4 mm to 32 ± 2.8 mm. The reason behind testing these bacterial and fungal species was that they are associated with many infectious diseases like pneumonia, meningitis, diarrhea, chronic lung disease, prostatitis, urinary-tract infections (UTI), wound infections and inter-abdominal infections. Our results are also coherent with the previous findings of Priyadarshi et al. [68] who reported insignificant antibacterial activity of *T. glaberrima* against *E. coli*. Similarly, Noreen et al. [69] also reported antibacterial potential in *T. glaberrima* methanolic extract against different bacterial strains. However, antimicrobial activity of *S. papilionacea* and *V. stocksii* has been reported for the first time. The antimicrobial property of flavonoids increases due to the existence of hydroxyl groups at particular sites in aromatic rings, while methylation declines the activity [70]. Hence, it can be inferred that the methylated flavonoids present in the methanolic extracts may be responsible for moderate antimicrobial activity.

RETRACTED

Furthermore, present study showed the existence of different volatile compounds in *T. glaberrima* and *V. stocksii* using GC-MS analysis for the first time. The investigation of various hydrocarbons and volatile compounds could help to verify the rationale behind the use of the plants as a cure for these diseases. Eicosane was recorded in highest concentration (44.60%) in *T. glaberrima* while 9,12-octadecadienoic acid (Z, Z)- was present in highest concentration (40.96%) in *V. stocksii.* In a nutshell, this is the first report demonstrating the biological potential of selected species and results revealed potential for optimization and application of polar extracts for the treatment of oxidative stress related diseases and/or that lead to the cancer-related deaths. Extracts of *S. papilionacea* and *T. glaberrima* are biologically active due to the presence of maximum number of bioactive compounds as compared to the *V. stocksii* extracts. Thus, logical extension via detailed *in vivo* study is recommended further to authenticate the validity of biological potential of these extracts.

## 5. Conclusion

This is the first study that provide detailed insight into the biological and biochemical properties of selected species, suggesting that the methanolic extracts possess strong antioxidant and anticancer activities that could be exploited in food and herbal industries. However, further studies are required for in-depth screening of phytochemicals and identification of active compounds that are associated with biological activities. Simultaneously, efforts should be made to conduct possible clinical studies to validate their toxicity potential so that best alternative herbal products could be formulated as a substitute of presently used man-made drugs.

## Figures and Tables

**Figure 1:** FTIR spectra indicating the presence of various functional groups (a) *S. papilionacea* (b) *T. glaberrima* (c) *V. stocksii.*

**Figure 2:** Total phenolic and flavonoid contents observed in five different extracts of *S. papilionacea*, *T. glaberrima* and *V. stocksii*. Data represents the mean of three replicates and each letter (a-h) indicates significance at *P* < 0.05.

**Figure 3:** Antioxidant assays of different extracts of *S. papilionacea*, *T. glaberrima* and *V. stocksii*. Data represents the mean of three replicates and standard deviation is indicated by the error bars (a) Total reducing power assay (b) CUPRAC assay (c) Total antioxidant capacity (d) DPPH radical scavenging assay.

RETRACTED

**Figure 4:** Pearson correlation analysis of antioxidant assays and phytochemicals (a) Total reducing power assay and phytochemical contents (b) CUPRAC assay and phytochemicals (c) Total antioxidant capacity and phytochemicals (d) DPPH radical scavenging assay of methanolic and chloroform extracts of three species and phytochemicals (r = Correlation coefficient).

**Figure 5:** Percentage viabilities observed in different extracts of *S. papilionacea*, *T. glaberrima* and *V. stocksii* against (a) HepG2 and (b) HT144 cells in comparison to the control. Pearson correlation analysis of phytochemicals with (c) HepG2 cell lines assay and (d) HT144 cell lines assay. Data represents the mean ± SD of two independent experiments and each letter (a-i) indicates significant difference at *p* < 0.05 as determined by LSD using statistix 8.1. ‘r' represents correlation co-efficient.

**Figure 6:** Chromatograms indicating the presence of total identified compounds (TIC) eluted at different retention times in the selected species (a) *T. glaberrima* (b) *V. stocksii.*

**Table 1:** PXR activation and CYP3A4 enzyme inhibition observed in cancer cell lines after treating with selected plant extracts.

Plant extracts	Fold increase in PXR at different concentrations			Inhibition of CYP3A4 enzyme [IC_50_ value (*μ*g/mL)]
	60 *μ*g/mL	20 *μ*g/mL	6.7 *μ*g/mL	
*S. papilionacea*	2.29 ± 0.20	1.47 ± 0.33	1.19 ± 0.28	27.5 ± 0.50
*T. glaberrima*	3.49 ± 0.34	1.98 ± 0.32	1.25 ± 0.15	15.0 ± 3.00
*V. stocksii*	2.70 ± 0.42	1.93 ± 0.40	1.28 ± 0.35	26.5 ± 1.50
Concentrations used for standard	**10 *μ*M**	**3.3 *μ*M**	**1.1 *μ*M**	
Fold induction by standard	2.70 ± 0.42	2.12 ± 0.15	1.89 ± 0.08	0.008 ± 0.001

Data represents mean ± SD (n = 2). Rifampicin was used as a positive control for PXR assay and Ketoconazole was used as a positive control for CYP_3_A_4_ enzyme inhibition assay. IC_50_ values were calculated using Graphpad Prism software.

**Table 2:** IC_50_ values and selectivity indices of selected plant extracts tested against malarial parasites.

Plant extracts	*P. Falciparum* D6		*P. Falciparum* W2		VERO
	IC_50_	SI	IC_50_	SI	IC_50_
*S. papilionacea*	> 47600	1	> 47600	1	> 47600
*T. glaberrima*	> 47600	1	> 47600	1	> 47600
*V. stocksii*	> 47600	1	> 47600	1	> 47600

IC_50_: 50% inhibitory concentration; SI: Selectivity indices.

**Table 3:** Inhibition zones determined by the antibacterial and antifungal activity of selected methanolic plant extracts.

Plant extracts	ZOI (mm) observed against bacterial strains		ZOI (mm) observed against fungal strains		
	*Escherichia coli*	Vancomycin-resistant *enterococcus faecium*	*Candida albicans*	*Cryptococcus neoformans*	*Aspergillus fumigatus*
*S. papilionacea*	8 ± 2.8	0 ± 0	12 ± 2.8	32 ± 2.8	2 ± 0
*T. glaberrima*	9 ± 0	11 ± 1.4	12 ± 1.4	22 ± 1.4	4 ± 2.1
*V. stocksii*	10 ± 0.7	2 ± 0	13 ± 1.4	29 ± 3.5	3 ± 1.4
Standard	29 ± 1.5	28 ± 1.8	30 ± 1.5	32 ± 2.7	28 ± 2.0

Data represents means ± SD (n = 2) and bacterial species which remain completely inactive (*P. aeruginosa*, *K. pneumoniae* and methicillin-resistant *S. aureus*) against selected extracts are not presented in the table. Oxytetracycline was used as a standard for antibacterial activity and chloramphenicol was used for antifungal activity; ZOI: zone of inhibitions.

RETRACTED

**Table 4:** Concentration (%) of compounds identified in *T. glaberrima* and *V. stocksii* at different retention times by using GC-MS method.

RT	Names of compounds	Molecular weight	Concentration (%)	
			*T. glaberrima*	*V. stocksii*
7.18	Heptane	100.125	0.575	1.176
46.24	2-Pentadecanone, 6,10,14-trimethyl-	268.277	0.378	0.388
46.4	Neophytadiene	278.297	13.226	5.274
46.66	2-Hexadecene, 3,7,11,15-tetramethyl-, [R-[R∗,R∗-(E)]]-	280.313	1.626	0.614
47.01	Cyclohexanol, 1-ethynyl-	124.089	2.294	0.605
47.47	3-Eicosyne	278.297	—	1.517
47.48	1-Tridecyne	180.188	3.951	—
48.48	Dibutyl phthalate	278.152	—	0.654
48.9	n-Hexadecanoic acid	256.240	3.858	16.096
49.87	Acetic acid, 2-[4-(4-oxo-2-thioxothiazol-5-ylidenemethyl)phenoxy]-, ethyl ester	256.096	—	0.465
52.10	9,12-Octadecadienoic acid, methyl ester, (E,E)-	294.256	—	0.318
52.91	9,12-Octadecadienoic acid (Z,Z)-	280.240	3.214	17.501
52.98	9,12,15-Octadecatrienoic acid, (Z,Z,Z)-	278.225	2.444	—
53.08	9,12-Octadecadienoic acid (Z,Z)-	280.240	5.582	23.464
57.03	Nonadecane	268.313	0.972	—
57.59	4,8,12,16-Tetramethylheptadecan-4-olide	324.303	—	0.719
59.31	Cyclotrisiloxane, hexamethyl-	222.056	0.498	0.754
60.05	1-methyl-4-phenyl-5-thioxo-1,2,4-triazolidin-3-one	207.047	1.933	—
60.45	Cyclotrisiloxane, hexamethyl-	222.056	0.475	—
61.01	Hexadecane	266.266	0.812	—
61.21	Tetrasiloxane, decamethyl-	310.127	0.482	—
61.21	Bis(2-ethylhexyl) phthalate	390.277	—	1.237
61.60	Tetrasiloxane, decamethyl-	310.127	—	0.693
62.53	Tetracosane	338.391	—	5.243
62.88	Cyclotrisiloxane, hexamethyl-	222.056	2.371	—
64.87	Nonadecane	268.313	3.984	—
67.13	Cyclotrisiloxane, hexamethyl-	222.056	0.429	—
68.64	Cyclotrisiloxane, hexamethyl-	222.056	—	1.286
67.89	2-Hydroxy-4-methoxybenzaldehyde, butyl ether	208.110	—	5.664
69.77	Eicosane	282.329	12.849	—
72.90	Cyclotrisiloxane, hexamethyl-	222.056	1.813	1.737
73.05	Cyclotrisiloxane, hexamethyl-	222.056	0.772	1.664
75.47	Cyclotrisiloxane, hexamethyl-	222.056	2.809	2.116
76.68	Cyclotrisiloxane, hexamethyl-	222.056	—	4.395
76.70	Eicosane	282.329	31.757	—
76.88	Cyclotrisiloxane, hexamethyl-	222.056	—	0.739
**Total identified compounds (TIC)**			99.104	94.319

∗Compounds are mentioned as detected from minimum to maximum retention time; RT: Retention time.

RETRACTED

## Data Availability

The data used to support the findings of this study are available from the corresponding author upon request.
